This article has been retracted.

# Rehabilitation of Post-Stroke Swallowing Dysfunction with Repeated Transcranial Magnetic Stimulation RTMS Based on Tomographic Images

**DOI:** 10.1155/2022/1118745

**Published:** 2022-09-13

**Authors:** Jin Liu, Hengye Zhuo, Mingliang Sun

**Affiliations:** ^1^Rehabilitation Department, Jiangsu Shuyang County Traditional Chinese Medicine Hospital, Suqian 223600, Jiangsu, China; ^2^Neurosurgery, Jiangsu Shuyang County Traditional Chinese Medicine Hospital, Suqian 223600, Jiangsu, China

## Abstract

In order to study the rehabilitation of dysphagia after stroke, this paper uses tomographic imaging technology and repeated transcranial magnetic stimulation rTMS therapy to verify the effect of this treatment method on the rehabilitation of dysphagia after stroke. In this study, the method of systematic review and meta-analysis are used to comprehensively collect the current published literature on the application of repeated transcranial magnetic stimulation in post-stroke dysphagia, and to quantitatively synthesize and qualitatively analyze the data and opinions. This article aims to explore the therapeutic effect and mechanism of repeated transcranial magnetic stimulation in the treatment of dysphagia after stroke, and to evaluate its effectiveness, so as to better guide the application of repetitive transcranial magnetic stimulation in the rehabilitation of dysphagia after stroke. The evaluation methods of rTMS for the clinical efficacy of PAS, FDS, VDS, DOSS, DD, and BI in patients with dysphagia after stroke are consistent. The influencing factors of rTMS on the swallowing function impairment of stroke include the choice of stimulation frequency, stimulation site, and stimulation time. Low-frequency stimulation of the contralateral hemisphere and high-frequency stimulation of the affected brain can reduce the excitability of the contralateral brain and enhance the excitability of the affected brain. The stimulation site is mainly in the pharyngeal cortex. Experiments show that rTMS can improve swallowing dysfunction after stroke within 2 weeks, and rTMS has no obvious side effects on swallowing dysfunction in patients with cerebral infarction.

## 1. Introduction

Due to the improvement of living standards and changes in living environment, the incidence of stroke has been increasing. In the comparison between urban and rural areas, the incidence in urban areas is slightly higher than that in rural areas. Dysphagia after stroke is a clinical symptom. It is caused by bleeding or blockage of blood vessels in the brain that damages the centers involved in swallowing, other secondary centers, or afferent and efferent nerves, thereby impairing one or more stages of swallowing, which makes it difficult for the patient to eat. About 37%–78% of stroke patients have dysphagia (dysphagia, choking on drinking water, tongue muscle weakness, drooling and others), which occurs in the oral and pharyngeal phases. This not only affects the quality of life of patients, but also causes aspiration, aspiration pneumonia, malnutrition, and ignorance of the order of diet. In the case of dysphagia in the chronic recovery phase, targeted rehabilitation can be performed. For patients with dysphagia after stroke, evaluation should be performed at the early stage (such as repeated salivary swallowing test, Kubota drinking test, examination of swallowing reflex, cough reflex). If there are obvious symptoms, it should be intervened as soon as possible. And reasonable dietary guidance should be given to patients who cannot eat, so as to reduce the complications caused by the inability to eat, thereby improving their quality of life. The application of repeated transcranial magnetic stimulation (rTMS) in the field of stroke rehabilitation is a research that has only emerged in recent years. Its studies on limb motor dysfunction, cognitive dysfunction, anxiety and depression and psychological disorders have been reported. However, there are relatively few studies on the treatment of dysphagia after stroke.

Research into the rehabilitation of swallowing dysfunction is ongoing. Atteya et al. systematically reviewed the studies evaluating the impact of physical therapy interventions on orofacial dysfunction after stroke [1]. Yu et al. demonstrated the application of electroacupuncture stimulation to patients with dysphagia and post-stroke constipation [2]. Peng et al. discussed the effect of early targeted rehabilitation training on the improvement of intonation and swallowing function of patients [3]. Hgglund et al. aimed to describe and analyze the relationship between dysphagia and malnutrition risk in older adults in short-term care [4]. Yhc et al. aimed to explore the mechanisms, risk factors, and clinical assessment of swallowing dysfunction and its associated symptoms [5]. Atsushi et al. aimed to evaluate dysphagia in patients with spinal cord and bulbar muscle atrophy [6]. This type of research cannot provide an intuitive image reference, so it needs to use tomographic images to achieve.

Some scholars have studied the tomographic images. Pietrzycka et al. evaluated the accuracy of determining the length of a tooth's root canal using preexisting cone beam computed tomography images [7]. Frank et al. used deep learning algorithms to automatically segment cone beam computed tomography images and detect periapical lesions [8]. This type of research is only at the theoretical level, and has not applied tomographic images to actual clinical research. Therefore, this study combines the two modules of tomographic image and swallowing dysfunction rehabilitation to realize the research on the rehabilitation of swallowing dysfunction after stroke based on repeated transcranial magnetic stimulation rTMS therapy based on tomographic images.

In this study, 315 literature are preliminarily screened by using the literature database, and 10 of them are different in the measurement indicators of rTMS on the swallowing function impairment after stroke, which are limited to qualitative ones, and the remaining 13 are included in the meta-analysis. The results show that the comprehensive impact scale SMD is 0.64, *P* < 0.00001, and there is a significant difference between the two. The results also show that with BI as the evaluation standard, the efficacy of rTMS on swallowing dysfunction after stroke is better than that of the control group.

## 2. Repeated Transcranial Magnetic Stimulation RTMS Therapy

The swallowing reflex process is shown in Figure 1 [9, 10].

This paper explains the role of tomographic images in this research by explaining the principle of 3D modeling of tomographic images [11, 12]. It is assumed that point (Ξ′, Ω′, Θ′) is obtained from point (Ξ, Ω, Θ) after moving distances ϱΞ, ϱΩ, and ϱΘ in the Ξ, Ω, and Θ axis directions respectively, as shown in Figure 2, the relationship between its coordinates is:

(1) $$\begin{array}{c} \left\{\begin{array}{c} \Xi^{\prime }=\Xi +\varrho \Xi \\ \Omega^{\prime }=\Omega +\varrho \Omega \\ \Theta^{\prime }=\Theta +\varrho \Theta \end{array}\right.\text{.} \end{array}$$

It can be expressed in matrix form as:

(2) $$\begin{array}{c} \left[\begin{array}{c} \Xi^{\prime }\\ \Omega^{\prime }\\ \Theta^{\prime } \end{array}\right]=\left[\begin{array}{ccc} 1 & 0 & 0\\ 0 & 1 & 0\\ 0 & 0 & 1 \end{array}\right]\left[\begin{array}{c} \Xi \\ \Omega \\ \Theta \end{array}\right]+\left[\begin{array}{c} \varrho \Xi \\ \varrho \Omega \\ \varrho \Theta \end{array}\right]\text{.} \end{array}$$

By setting point (Ξ, Ω, Θ) to be scaled and transformed, point (Ξ′, Ω′, Θ′) can be obtained, as shown in Figure 3, the coordinate relationship between the two points is:

(3) $$\begin{array}{c} \left\{\begin{array}{c} \Xi^{\prime }=\Lambda_{\Xi }\Xi \\ \Omega^{\prime }=\Lambda_{\Omega }\Omega \\ \Theta^{\prime }=\Lambda_{\Theta }\Theta \end{array}\right.\text{.} \end{array}$$

Among them, Λ_Ξ_, Λ_Ω_, and Λ_Θ_ are the enlargement or reduction ratios along the Ξ, Ω, and Θ axes, respectively [13, 14]. The matrix form is:

(4) $$\begin{array}{c} \left[\begin{array}{c} \Xi^{\prime }\\ \Omega^{\prime }\\ \Theta^{\prime } \end{array}\right]=\left[\begin{array}{ccc} \Lambda_{\Xi } & 0 & 0\\ 0 & \Lambda_{\Omega } & 0\\ 0 & 0 & \Lambda_{\Theta } \end{array}\right]\left[\begin{array}{c} \Xi \\ \Omega \\ \Theta \end{array}\right]\text{.} \end{array}$$

In the three-dimensional coordinate system, by setting the given coordinate (Ξ, Ω, Θ)=(*𝔄* cos *𝔅*, *𝔄* sin *𝔅*, Θ) and using the right helix rule, after rotating *ℭ* angles around the Θ axis, (Ξ′, Ω′, Θ′) can be obtained, as shown in Figure 4 [15, 16].

(5) $$\begin{array}{c} \left\{\begin{array}{c} \Xi^{\prime }=\Xi \;\cos\;C-\Omega \;\sin\;C\\ \Omega^{\prime }=\Xi \;\sin\;C+\Omega \;\cos\;C\\ \Theta^{\prime }=\Theta \end{array}\right.\text{.} \end{array}$$

The matrix form is:

(6) $$\begin{array}{c} \left[\begin{array}{c} \Xi^{\prime }\\ \Omega^{\prime }\\ \Theta^{\prime } \end{array}\right]=\left[\begin{array}{ccc} \cos\;C & -\sin\;C & 0\\ \sin\;C & \cos\;C & 0\\ 0 & 0 & 1 \end{array}\right]\left[\begin{array}{c} \Xi \\ \Omega \\ \Theta \end{array}\right]\text{.} \end{array}$$

The formula around Ω axis is:

(7) $$\begin{array}{c} \left[\begin{array}{c} \Xi^{\prime }\\ \Omega^{\prime }\\ \Theta^{\prime } \end{array}\right]=\left[\begin{array}{ccc} \cos\;D & 0 & \sin\;D\\ 0 & 1 & 0\\ -\sin\;D & 0 & \cos\;D \end{array}\right]\left[\begin{array}{c} \Xi \\ \Omega \\ \Theta \end{array}\right]\text{.} \end{array}$$

The formula around the Ξ axis is:

(8) $$\begin{array}{c} \left[\begin{array}{c} \Xi^{\prime }\\ \Omega^{\prime }\\ \Theta^{\prime } \end{array}\right]=\left[\begin{array}{ccc} 1 & 0 & 0\\ 0 & \cos\;E & -\sin\;E\\ 0 & \sin\;E & \cos\;E \end{array}\right]\left[\begin{array}{c} \Xi \\ \Omega \\ \Theta \end{array}\right]\text{.} \end{array}$$

The composite rotation matrix is represented as:

(9) $$\begin{array}{c} o\left(C\right)=t^{-1}*o_{\Xi }^{-1}\left(E\right)*o_{\Omega }^{-1}\left(D\right)*o_{\Theta }\left(C\right)*o_{\Omega }\left(D\right)*o_{\Xi }\left(E\right)*t\text{.} \end{array}$$

Among them, the translation matrix is:

(10) $$\begin{array}{c} t=\left[\begin{array}{ccc} 1 & 0 & \begin{array}{cc} 0 & -\Xi_{1} \end{array}\\ 0 & 1 & \begin{array}{cc} 0 & -\Omega_{1} \end{array}\\ \begin{array}{c} 0\\ 0 \end{array} & \begin{array}{c} 0\\ 0 \end{array} & \begin{array}{c} \begin{array}{cc} 1 & -\Theta_{1} \end{array}\\ \begin{array}{cc} 0 & 1 \end{array} \end{array} \end{array}\right]\text{.} \end{array}$$

The rotation matrices are:

(11) $$\begin{array}{c} \begin{array}{c} o_{\Theta }\left(C\right)=\left[\begin{array}{ccc} \cos\;C & -\sin\;C & \begin{array}{cc} 0 & 0 \end{array}\\ \sin\;C & \cos\;C & \begin{array}{cc} 0 & 0 \end{array}\\ \begin{array}{c} 0\\ 0 \end{array} & \begin{array}{c} 0\\ 0 \end{array} & \begin{array}{c} \begin{array}{cc} 1 & 0 \end{array}\\ \begin{array}{cc} 0 & 1 \end{array} \end{array} \end{array}\right]\\ o_{\Omega }\left(D\right)=\left[\begin{array}{ccc} \cos\;D & 0 & \begin{array}{cc} \sin\;D & 0 \end{array}\\ 0 & 1 & \begin{array}{cc} 0 & 0 \end{array}\\ \begin{array}{c} -\sin\;D\\ 0 \end{array} & \begin{array}{c} 0\\ 0 \end{array} & \begin{array}{c} \begin{array}{cc} \cos\;D & 0 \end{array}\\ \begin{array}{cc} 0 & 1 \end{array} \end{array} \end{array}\right]\\ o_{\Xi }\left(E\right)=\left[\begin{array}{ccc} 1 & 0 & \begin{array}{cc} 0 & 0 \end{array}\\ 0 & \cos\;E & \begin{array}{cc} -\sin\;E & 0 \end{array}\\ \begin{array}{c} 0\\ 0 \end{array} & \begin{array}{c} \sin\;E\\ 0 \end{array} & \begin{array}{c} \begin{array}{cc} \cos\;E & 0 \end{array}\\ \begin{array}{cc} 0 & 1 \end{array} \end{array} \end{array}\right] \end{array}\text{.} \end{array}$$

The vector value of the sight direction in the object coordinate system is set to (cos *𝔈*, cos *𝔇*, cos *𝔉*), and the sight direction is set to the Θ-axis direction, then the object coordinate is transferred to the transformation matrix of the image coordinate, and *ℴ* in *ℴ* · *𝓉* is:

(12) $$\begin{array}{c} {o=o}_{\Omega }\left(D\right)\cdot o_{\Xi }\left(E\right)\text{.} \end{array}$$

For parallel projection (as shown in Figure 5):

(13) $$\begin{array}{c} 0<\Xi <1,0<\Omega <1,0<\Theta <1\text{.} \end{array}$$

It is assumed that the start and end points of the line segment are *𝔑*_0_(Ξ_0_, Ω_0_, Θ_0_) and *𝔑*_1_(Ξ_1_, Ω_1_, Θ_1_), respectively, the formula of the line can be expressed in parametric form as:

(14) $$\begin{array}{c} \left\{\begin{array}{c} \Xi =\Xi_{0}+\left({\Xi_{1}-\Xi }_{0}\right)X\\ \Omega =\Omega_{0}+\left({\Omega_{1}-\Omega }_{0}\right)X\\ \Theta =\Theta_{0}+\left({\Theta_{1}-\Theta }_{0}\right)X \end{array}\right.\text{.} \end{array}$$

When the line segment and the boundary surface of the viewport are intersected, then

(15) $$\begin{array}{c} 1=\Omega_{0}+\left({\Omega_{1}-\Omega }_{0}\right)X^{\prime }\text{.} \end{array}$$

Thereby

(16) $$\begin{array}{c} X^{\prime }=\frac{1-\Omega_{0}}{{\Omega_{1}-\Omega }_{0}}\text{ .} \end{array}$$

By putting *𝔛*′ into the parametric equation, the coordinates of the intersection can be obtained [17, 18].

The CT value of the CT image reflects the tissue's absorption of *X*-rays (the attenuation coefficient is *𝔜*):

(17) $$\begin{array}{c} S=\frac{T*\left(Y-Y_{v}\right)}{Y_{v}}\text{.} \end{array}$$

Among them, *𝔜*_*𝔳*_ is the *X*-ray attenuation coefficient of water, and *𝔗* is a constant, which is mostly taken as 1000.

### 2.1. Meta of RTMS Therapy on the Recovery of Swallowing Dysfunction after Stroke

Inclusion criteria: patients who meet the World Health Organization's definition of stroke and are diagnosed with stroke (ischemic or hemorrhagic) with dysphagia by clinically relevant examinations (CT or MRI); patients who have obvious clinical symptoms and signs, mainly manifested as dysphagia, orofacial muscle and tongue muscle apraxia, and have the existence of dysphagia confirmed by the evaluation of the water drinking test, the dysphagia scale, or the TV *X*-ray swallowing function test (VFSS), and other methods; patients who voluntarily participate in clinical research and signing of informed consent [19, 20].

Exclusion criteria: dysphagia not caused by stroke or apraxia of muscles related to swallowing; patients with long-term nasogastric feeding tube or esophagostomy; in pregnancy; history of epilepsy or other central nervous system diseases; patients with metal objects in the brain or metal built-in in the body, such as pacemakers, nerve stimulators, drug pumps, cochlear implants, and so on; patients with the existence of serious medical diseases; patients with the inability to cooperate with the completion of clinical research due to cognitive impairment and mental illness.

Intervention (I): in the experimental group, planned and organized rTMS therapy was administered to enrolled patients. The stimulation frequency (low frequency or high frequency), stimulation intensity, stimulation site, stimulation time, course of treatment, and others were not limited. In the control group, the enrolled patients were treated with rTMS with no effect or placebo effect. Treatment parameters should be consistent with the experimental group and be either ineffective or placebo-responsive.

Control measures (C): the control group can be treated with placebo, conventional rehabilitation treatment, and blank treatment.

Outcome index (O): PAS represents penetration-aspiration scale score; FDS represents functional dysphagia scale score; VDS represents television fluoroscopy dysphagia scale score; DOSS represents dysphagia outcome and severity score; DD represents dysphagia severity classification; Barthel Index represents Barthel index score.

Through the preliminary screening of the literature database, 315 literature (173 in Chinese and 142 in English, as shown in Figure 6) are obtained. After screening for repeated publications, excluding unsuitable research themes and reviews, a total of 23 studies are included, including 23 in English and 0 in Chinese. Among them, 10 literature have different measurement indicators for rTMS in the treatment of post-stroke dysphagia, which cannot be analyzed quantitatively, but can only be analyzed qualitatively, and the remaining 13 literature are included for meta-analysis.

The general characteristics of the included literature are shown in Table 1.

The types of stroke in the literature are shown in Table 2.

Table 2 shows that a total of 277 subjects are included, 163 in the treatment group and 114 in the control group. The number of ischemic strokes in the experimental group is 107.

Seven studies use rTMS and sham control, two studies use rTMS with other treatments (pharyngeal electrical stimulation, traditional treatment of dysphagia), one study uses rTMS and rTMS control, and three studies use their own before and after control. The shortest course of treatment is 5 days and the longest is 6 weeks. The number of people in different frequency stimulation groups is shown in Table 3.

Table 3 shows 52 cases in the 1 Hz treatment group, 39 cases in the 3 Hz treatment group, and 24 cases in the 5 Hz treatment group. On the stimulation site, there are 24 cases in the bilateral cerebral hemisphere stimulation group, 67 cases in the contralateral hemisphere stimulation group, and 72 cases in the affected cerebral hemisphere.

In the included literature, seven randomized controlled trials use PAS as an outcome indicator, of which Kim2021 use two intervention methods of 1 Hz low frequency (in the pharyngeal cortex of the contralateral hemisphere) and 5 Hz high frequency (in the pharyngeal cortex of the affected hemisphere). Another four papers, Lim 2016, Lee 2015, Park 2017, and Park 2016, conducted a follow-up after the trial. There are three studies in the low-frequency group and eight studies in the high-frequency group. The meta-analysis results of the PAS score between the rTMS treatment group and the control group are shown in Figure 7.

In the data shown in Figure 7, the meta-analysis shows that the improvement of the PAS score of the experimental group is better than that of the control group, and the difference is statistically significant (*P*=0.0004 and *P*=0.0001). After the data are combined, the effect size SMD = −0.71, *P* < 0.00001, the difference is still statistically significant, indicating that rTMS is more effective than the control group when PAS is used as the outcome indicator for the treatment of dysphagia after stroke.

The meta-analysis results of the treatment group and the control group on the FDS score are shown in Table 4.

In the included literature, four RCTs use BI as an outcome measure, and four studies are followed up. Among them, Du 2016 has 1 Hz and 3 Hz treatment groups, and they are followed up in the first, second, and third months, respectively. Khedr 2019 and Khedr 2020 are followed up in the first month and the second month, respectively, and there are 16 treatment groups and control groups. There are 164 cases in the treatment group and 150 cases in the control group. The meta-analysis results of the treatment group and the control group on the BI score are shown in Figure 8.

Figure 8 shows that the effect size SMD = 0.64, *P* < 0.00001 after the data is merged, the difference is still statistically significant. It is suggested that rTMS is more effective than the control group in the treatment of dysphagia after stroke when BI is used as the outcome indicator.

In the included literature, Two RCTs use DOSS as an outcome measure, both studies have a follow-up at the fourth week, and the Park 2016 treatment group has bilateral stimulation and unilateral stimulation. There are six treatment groups and control groups, including 68 cases in the treatment group and 68 cases in the control group. The meta-analysis results of the treatment group and the control group on the DOSS score are shown in Figure 9.

Figure 9 shows that the effect size SMD = 0.56, P=0.002 after the data is merged, the difference is still statistically significant. It is suggested that rTMS is more effective than the control group when DOSS is used as the outcome indicator in the treatment of dysphagia after stroke.

In the included literature, two RCTs use DD as an outcome measure, and both studies have a follow-up at the first and second months. Among them, Khedr 2020 has two groups of dorsolateral medulla oblongata (LMI) and other brainstem infarction (OBI), and the two groups are compared with each other. There are nine treatment groups and control groups, including 75 cases in the treatment group and 69 cases in the control group. The meta-analysis results of the treatment group and the control group on the DD score are shown in Figure 10.

Figure 10 shows that the effect size SMD = −4.09, *P* < 0.00001 after the data are merged, the difference is still statistically significant. It is suggested that rTMS is more effective than the control group in the treatment of dysphagia after stroke when DD is used as the outcome indicator.

The Meta-analysis results of the treatment group and the control group on the VDS score are shown in Table 5.

Table 5 shows that rTMS has no statistical difference when VDS is used as the outcome indicator in the treatment of dysphagia after stroke.

Reference [3] used 1 Hz rTMS, nerve and muscle electrical stimulation (NMES), and traditional dysphagia therapy (CDT) to compare the treatment of dysphagia after subacute unilateral stroke. The patients were given two types of food, semisolid, and liquid respectively. VFSS and different swallowing disorder scales assessed the final efficacy. The results showed a significant improvement in FDS and PAS in the rTMS and NMES groups compared with the CDT group when fluids were administered to the patients. However, there was no significant difference between the rTMS group and the NMES group. When patients were given semisolids, all three groups of patients improved on all measures, but there were no between-group differences.

Reference [2] used 1 Hz rTMS to stimulate the contralateral cerebral hemisphere to treat four cases of stroke patients with unilateral cerebral hemisphere damage. During the treatment, each patient was given traditional rehabilitation therapy 3 days a week for a total of 6 weeks. The evaluation metric was the Mann Swallowing Ability Assessment (MASA), which showed the greatest change in MASA scores at the end of the first week of treatment, with a rate of change of 35%. All four patients had resolution of dysphagia by the end of the second week of treatment.

Similarly, Reference [1] used 1 Hz rTMS to stimulate seven patients with unilateral hemisphere damage. The treatment time was 5 days, 20 minutes a day, and the swallowing index (DHI) was used as an index. The results showed that after the treatment, the scores of swallowing coordination, aspiration, and residual were improved better. But the oral transit time, pharyngeal transit time, and laryngeal closure time did not change much. The most significant changes occurred after treatment, and the effects lasted for at least 2 weeks. The results showed that the motor cortex, represented by the pharyngeal muscle, could regulate the progress and progression of swallowing, which could effectively reduce the residual amount of debris in the pharynx and aspiration.

Reference [4] also used 1 Hz, 3 Hz, and sham stimulation groups to treat patients with dysphagia after stroke. The 1 Hz group stimulated the unaffected side of the patient, and the 3 Hz group stimulated the affected side of the patient. The course of treatment was 5 days. The results showed that in terms of clinical dysphagia score, the treatment group, regardless of the 1 Hz group or the 3 Hz group, had significant improvement compared with the control group.

Reference [5] used 1 Hz and 5 Hz as the treatment groups, and the control group as the sham stimulation group. The 1 Hz group stimulated the affected side of the patient, and the 5 Hz group stimulated the healthy side of the patient. The course of treatment was 10 days. The results showed that the 1 Hz group had significant improvement in the three-scale evaluations, while the 5 Hz group had no significant improvement. The final conclusion was that low-frequency rTMS promoted the recovery of swallowing function in patients. In a recent study, inhibitory rTMS was used to stimulate the motor cortex of the pharyngeal muscle with the aim of demonstrating its role in regulating swallowing activity and demonstrating asymmetry in brain functional activity. When either side of the brain hemisphere was stimulated with inhibitory rTMS, it resulted in stronger responses that ultimately altered the number of normal and fast swallows.

Reference [7] used 3 Hz stimulation of the affected cerebral hemisphere as the treatment group, and sham stimulation as the control group. The patients with unilateral ischemic stroke were intervened. The degree of dysphagia (DD), Barthel index, motor evoked potential (MEP) and hand grasping ability were selected as outcome indicators. Follow-up was carried out at the first month and the second months. The results showed that the degree of dysphagia and Barthel index were affected in both the treatment group and the control group, and the time × group had significant significance. The grasping ability of the hand was only significantly improved in time, and improved in group and group × time, but it was not statistically significant. A scholar found that when rTMS was applied to the pharyngeal cortex of any hemisphere, the excitability of both cerebral hemispheres increased. This demonstrated the possibility that the recovery of the patients in the study was due to impulses from the corticobulbar tract to the swallowing center of the brainstem. This physiologic pattern of recovery differed from the observed natural recovery process, which found that patients with dysphagia after their first stroke had few synaptic-to-nerve connections in the affected hemisphere. However, the contralateral hemisphere increased excitability. From this, they concluded that recovery from dysphagia was different from recovery of hand function. The innervation of the hand was unilateral, while the swallowing function was bilateral, that was, the recovery of swallowing function depended on the increase of the output of the contralateral hemisphere.

Reference [8] used 3 Hz to intervene in two groups of patients with a specific type of stroke. One group consisted of 11 patients with dorsolateral medullary syndrome (LMI), and the other group consisted of 11 other types of brainstem infarction (OBI), of which 6 were true stimulation and 5 were sham stimulation in the LIM group. In the OBI group, 5 cases were true stimuli and 6 cases were sham stimuli. Because of the brainstem injury, the study used stimulation of bilateral esophageal cortical regions. All patients receiving true stimulation recovered swallowing function immediately after 5 days of treatment, and the effect lasted for at least 2 months. While patients with sham stimulation continued to have dysphagia until 2 months later. The final conclusion was that rTMS might be an effective adjuvant therapy for dysphagia caused by dorsolateral medullary syndrome and other types of brainstem infarction. The peculiarity of this study is that the lesions of the subjects are in the brainstem. The brainstem is the secondary center of swallowing, which receives the afferent nerve impulses from the bilateral cortex, and changes elements through the two swallowing centers in the medulla oblongata, the nucleus doubtful and the nucleus tractus solitarius. Then the efferent nerve impulses reach the swallowing muscles. The brainstem infarction is mostly in one side of the brainstem, so the recovery of swallowing function may be played by the premotor neurons in the contralateral hemisphere and the contralateral medulla oblongata after the swallowing center on one side is injured.

Reference [6] used 3 Hz combined with intensive swallowing rehabilitation training to treat four patients with dysphagia after stroke. All patients had bilateral cerebral infarction, and the intervention method was also bilateral intervention, that is, stimulation of bilateral pharyngeal cortex, but no training with food. The results showed that this combination therapy could improve the delay time of laryngeal elevation, improve the function of pharyngeal constrictor muscles, reduce the incidence of aspiration pneumonia by reducing the inhalation of saliva at night, improve the muscle strength of the tongue, coordinate the chewing process and reduce the occurrence of reflux esophagitis.

In Reference [13], nine patients with dysphagia after stroke were intervened with 5 Hz, and a control group of the same number was set up. The intervention method was performed using the contralateral cerebral cortex. The results showed that significant improvement in both VDS and PAS on imaging. High-frequency rTMS at 5 Hz stimulated the contralateral cerebral hemisphere. The theoretical basis was that when a stroke patient had an oropharyngeal dysphagia, the oropharyngeal cortex of the contralateral side had a certain functional relationship with the pharyngeal cortex. And the size of this cortical area gradually increased with the recovery of swallowing function.

Reference [11] used 5 Hz rTMS, pharyngeal electrical stimulation (PES), and paired combined stimulation (PAS) to explore the mechanism of improvement of dysphagia after stroke. The results showed that PES and PAS could beneficially regulate the excitability of the corticomedullary tract in the motor cortex of the pharyngeal muscle, and the function of the contralateral cerebral hemisphere was also improved accordingly. When comparing the true and sham groups, the true stimulation group reduced aspiration by 15%. In rTMS group, there was no significant difference between true stimulation and sham stimulation in improving cortical excitability and cumulative score of penetration-aspiration. Interestingly, both PES and PAS stimulation methods mainly used peripheral nerve afferent impulses, and both methods could increase the excitability of the affected hemisphere. The increase in PAS excitability mainly occurred immediately after the end of treatment, while the PES mainly occurred 30 minutes after the end of treatment. Therefore, it was reasonable to believe that the two modalities had different temporal and neurofiber recruitment mechanisms in enhancing bilateral interhemispheric cortical associativity. In the rTMS group, when the intervention was applied to the contralateral cerebral hemisphere, brain excitation was significantly increased in both the true and false stimulation groups. This suggested that sham stimulation might have some biological effect on cortical function. From the above results, it may be inferred that both PES and PAS using peripheral stimulation produce bilateral cortical effects, and a single rTMS application may not be sufficient to produce bilateral effects and improve functional outcomes. The final conclusion was that the improvement of swallowing function might be more caused by the improvement of the contralateral neural pathway.

Reference [9] used 5 Hz rTMS intervention in four patients with dysphagia after unilateral stroke, including two cases of true stimulation and two cases of sham stimulation. The purpose of its intervention was to investigate the short-term effects of rTMS at a frequency of 5 Hz. The location of the intervention was also different from other studies. The main stimulation point was the motor cortex of the tongue muscle on the affected side. The outcome indicators were the pressure of the tongue muscle (TP), the oropharyngeal swallowing efficiency (OPSE), and the swallowing-related quality of life questionnaire (SAPP). The results showed that patients in the true stimulation group had improvements in swallowing function and swallowing-related quality of life questionnaires, and this effect lasted for 1 week to 1 month after treatment. The improvement in OPSE made the patient's swallowing process more efficient and safer. Another benefit was that the patient could swallow effectively when encountering different shapes of food (including liquid, semi-liquid and paste) during the meal. Another positive finding of the study was that the quality of life of the patients in the true stimulation group was also improved, and the functional improvement after true stimulation could reduce the patient's self-perceived ability to swallow impaired swallowing.

Reference [12] used 10 Hz rTMS to intervene two groups of patients with dysphagia after stroke. The test group used the motor evoked potential threshold from the suprahyoid muscle group, and the control group used the motor evoked potential threshold from the abductor pollicis brevis. The results showed that there was a significant difference between the experimental group and the control group in the outcome indicators DOSS, and there was no significant difference between the experimental group and the control group in the outcome indicators PAS and FDS. Both were improved, but without statistically significant. The study delved into why the DOSS scale was statistically significant, but the PAS and FDS were not. The possible reason was that this study took the suprahyoid muscle group as the research object of swallowing disorder, which means that the pharyngeal phase of the swallowing process is the focus of attention. The FDS scale, as a tool to quantify the degree of dysphagia, assessed both the pharyngeal and oral phases, so the scale might not be too sensitive. The PAS scale mainly reflected the penetration of substances in the oral cavity into the airway during the VFSS examination. In this study, PAS was used to assess fluid status. Clinically, recovery of dysphagia is more easily observed when tested with solid food than with liquid food, so the PAS scale is less sensitive when dysphagia is predominantly solid food. The DOSS scale records the outcome of swallowing function and reflects the dietary status through objective assessment, so it can not only reflect the pharyngeal phase of the swallowing process but also reflect the improvement of solid food dysphagia. The suprahyoid muscle group is considered to be the target of dysphagia stimulation in this test. Dysphagia after stroke is mainly due to problems in the pharyngeal phase, that is, the reduction of larynx access to the functional activity of swallowing-related muscle groups. Two studies reported that electrical stimulation of the pharynx caused the sternohyoid and scapolohyoid muscles to contract to lower the position of the hyoid bone, which interfered with the swallowing process.

Reference [10] used 10 Hz rTMS as the intervention measure, and set up three groups of bilateral stimulation group, unilateral stimulation group, and sham stimulation group to control each other. The results showed that all four scales were statistically significant in terms of time × group. At the first follow-up, the improvement in scores on the four scales was statistically significant in the bilateral stimulation group compared with the unilateral stimulation combined with sham stimulation group. At the second follow-up, only the bilateral stimulation group had a statistically significant improvement over the other two groups in CDS scores. Ultimately, it was suggested that high-frequency bilateral stimulation of the mandibular hyoid cortex had a greater improvement in swallowing function than single contralateral stimulation.

## 3. Conclusion

This systematic review collects data from a clinical trial of continuous transcranial magnetic stimulation therapy in patients with post-stroke dysphagia. The data of possible combined studies are quantified, the studies that cannot be combined are qualitatively analyzed, and the effect of rTMS in the treatment of SRD is comprehensively evaluated. And the results are concluded that rTMS has a good clinical effect on posttreatment swallowing dysfunction, and the difference in effect can be sustained for a long time. The main problems of this paper are that the literature included are all in English, the quantity is small, and there are few researches on relevant aspects in China. In the included trials, the sample size is too small, the intervention time is in the acute phase, and the follow-up time is less than 3 months. The research directions of this paper include large multicenter samples, the expansion of the sample size, and the increase of research on various groups. According to the grade and stage of swallowing dysfunction, rTMS is used for different interventions to further improve the treatment plan of rTMS. In this paper, neurophysiology and imaging are combined to deeply explore the mechanism of rTMS on stroke swallowing dysfunction, and to explore its mechanism of action in order to seek better treatment methods.

## Figures and Tables

**Figure 1:** Process of swallowing reflex.

**Figure 2:** Panning.

**Figure 3:** Zoom.

**Figure 4:** Rotation.

**Figure 5:** Parallel projection.

**Figure 6:** Literature screening process and results.

**Figure 7:** Meta-analysis of PAS scores. *Note.* SMD represents standardized mean difference; weight represents the weight of each included study.

**Figure 8:** Meta-analysis of BI scores.

**Figure 9:** Meta-analysis of DOSS scores.

**Figure 10:** Meta-analysis of DD scores.

**Table 1:** Basic characteristics of included literature.

Numbering	Research	years	Type of study	Sample size
1	Verin	2019	SCT	6
2	Ghelichi	2016	SCT	5
3	Lim	2016	RCT	51
4	Du	2016	RCT	42
5	Kim	2021	RCT	29
6	Momosaki	2016	SCT	5
7	Khedr	2019	RCT	23
8	Khedr	2020	RCT	19
9	Cheng	2015	SCT	5
10	Park	2017	RCT	17
11	Michou	2016	RCT	15
12	Lee	2015	PDS	31
13	Park	2016	RCT	27

*Note.* RCT is a randomized controlled trial; SCT is a self-control before and after; PDS is a paired design study.

**Table 2:** Types of stroke.

Stroke type	Test group (cases)	Control group (case)	Total
Ischemic stroke	107	69	176
Hemorrhagic stroke	35	33	68
Not clear	21	12	33
Total	163	114	277

**Table 3:** Number of people in different frequency stimulation groups.

Frequency	1 Hz	3 Hz	5 Hz	10 Hz
Number of cases	52	39	24	51
Stimulation site	Bilateral	Healthy side	Affected side	
Number of cases	24	67	72	

**Table 4:** Meta-analysis of FDS scores.

Study	Weight (%)	SDM	*P* Value
Kim 2021	28.7	−0.285	0.003
Lim 2016	37.8	−0.77	0.09
Lee 2015	33.5	−0.645	0.0008

**Table 5:** Meta-analysis of VDS scores.

Study	Weight (%)	SDM	*P* Value
Kim 2021 high	21.1	0.11	0.53
Kim 2021 low	18.4	0.98	0.53
Lim 2016 2 week	30.0	0.38	0.53
Lim 2016 4 week	30.5	0.18	0.53

## Data Availability

No data were used to support this study.
